# NRXN2 Possesses a Tumor Suppressor Potential via Inhibiting the Growth of Thyroid Cancer Cells

**DOI:** 10.1155/2021/7993622

**Published:** 2021-11-03

**Authors:** Cui Ma, Youyou Zhang

**Affiliations:** ^1^Department of Endocrinology, Liangzhu Hospital, Moganshan Road, Hangzhou, Zhejiang, China 311113; ^2^Department of Endocrinology, First People's Hospital of Taizhou Affiliated Wenzhou Medical University, Hengjie Road, Taizhou, China 318020

## Abstract

Thyroid cancer (THCA) is a common endocrine malignant tumor, and its global incidence of THCA has increased significantly. Neurexin 2 (NRXN2) is involved in the progression of some diseases. Nevertheless, it is still elusive towards the clinical implication and function of NRXN2 in THCA. As The Cancer Genome Atlas (TCGA) data demonstrated, we conducted a study to explore the links between NRXN2 expression and clinical features. Additionally, our data exhibited that, compared to normal thyroid tissues, NRXN2 showed low expression in THCA tissues. 20 important genes associated with NRXN2 were screened and identified. KEGG analysis data displayed that NRXN2 exhibited a link to the neuronal system, insulin secretion modulation, energy metabolism integration, muscle contraction, cardiac conduction, and neural adhesion molecule 1 (NCAM1) interactions. Our results in depth affirmed that NRXN2 was decreased in the tissues and cell lines of THCA patients. Functionally, we proved that overexpressing NRXN2 resulted in an inhibition of THCA cell proliferation, migration, and invasion *in vitro*. Collectively, our study demonstrated that, for the first time, NRXN2 behaved as an inhibitor of neoplasm and a promising biomarker in THCA.

## 1. Introduction

In the past 30 years, the global incidence of thyroid cancer (THCA) has increased significantly, mainly due to the increase in papillary thyroid cancer (PTC) [1, 2]. THCA is a common endocrine malignant neoplasm, but its prognosis is satisfying [3]. Therefore, the incidence of THCA has increased rapidly, but the lethality ratio remains flat [4]. For low-risk THCA, this reduction in the degree of treatment involves the degree of surgery, including total thyroidectomy, lobectomy, or surgery without active monitoring, and also, indications of radioactive iodine (RAI) involved are used [5]. Dosage and stimulation method, indications of inhibitory thyroxine therapy, and the scope and method of follow-up should be adapted to the risk of recurrence. Molecular marker tests may help guide customized treatments for patients with thyroid nodules and THCA [6]. Preoperative risk stratification using molecular markers can also be applied to better detect the most favorable scope of thyroidectomy for THCA patients [6].

Neurotoxins belong to a family of presynaptic unidirectional transmembrane proteins, displaying as organizers of synapses in mammals. Neurotoxin comprises three genes NRXN1, NRXN2, and NRXN3. Each of the three genes generates two forms: a longer *α*-form and a shorter *β*-form. The alterations of the NRXN gene are reported in various neuropsychiatric diseases, containing autism spectrum disorder (ASD), schizophrenia, intellectual disability (ID), and addiction [7]. NRXN2 has been initially explored in tumors. One study reported that NRXN2 negatively regulated the activity of nuclear factor erythroid 2-related factor 2 (NRF2) and participates in the emergence and progression of multiple diseases, like carcinoma, metabolism, and neurodegenerative diseases [8]. One study identifies NRXN2 as a reliable predictor of overall survival in medulloblastoma [9], which is conducive to well understand medulloblastoma's pathogenesis and treatment in the future. Another study shows that the deletion of the gene NRXN2 has been described to be involved in synaptogenesis, dendritic branching, and multiple endocrine neoplasia type 1 [10]. Our findings imply that NRXN2 plays essentially in some carcinomas. Till now, there is little known on NRXN2's clinical signification and function in THCA.

Here, based on TCGA database, the difference in NRXN2 expression between THCA and nontumor tissues was identified. Through KEGG analysis, we explored the possible role of NRXN2 in the tumorigenesis of THCA. The association existing in NRXN2 expression and clinicopathological features or overall survival was analyzed using TCGA dataset. Through GSEA analysis, we identified the relationship between NRXN2 and the antitumor function of specific immune cells. qRT-PCR was taken to measure NRXN2 mRNA expression in THCA tissues and cell lines. Then, we conducted the CCK-8 assay and Transwell assay to explore the influence of NRXN2 on THCA cell proliferation, cell migration, and invasion. All of these results suggested that NRXN2 functioned as a tumor suppressor gene and could serve as a novel target for THCA therapy.

## 2. Materials and Methods

### 2.1. Analysis of NRXN2 Gene Expression

The original RNA sequencing dataset and the clinical features of TCGA-THCA column could be downloaded from The Cancer Genome Atlas (TCGA) website (https://cistrome.shinyapps.io/timer/). TCGA data was exploited to analyze the mRNA level of NRXN2 in THCA.

### 2.2. Analysis of Gene Set Enrichment

The Molecular Signatures Database (MSigDB, https://www.gsea-msigdb.org/gsea/msigdb/index.jsp) is a collection of annotated gene sets used in Gene Set Enrichment Analysis (GSEA) software. MSigDB contains annotated gene sets involving biochemical pathways, signal cascades, expression profiles of research publications, and other biological concepts. GSEA is a calculation method used to assess whether a set of a priori defined genes shows statistically significant and consistent differences between two biological states. We used immunologic signature gene sets from the MSigDB database to analyze the correlation between the expression level of NRXN2 and tumor-infiltrating immune cells.

### 2.3. Analysis of Pathways

The Database for Annotation, Visualization, and Integrated Discovery v6.8 (DAVID, https://david.ncifcrf.gov/home.jsp) was employed to conduct the KEGG pathway enrichment analysis. Notably, top results with the FDR ≤ 0.05 were identified. The enrichment pathway and process are demonstrated in Figure 1, where the *x*-axis and *y*-axis represented the abundance ratio records in the database and the enrichment of all functional category ratio.

### 2.4. Clinical Samples

35 THCA tissues and paired adjacent normal tissues were obtained from surgical patients in First People's Hospital of Taizhou Affiliated Wenzhou Medical University. All patients did not receive any chemical or physical treatment prior to operation. All tissues were defined as THCA after pathological examination, followed by putting in liquid nitrogen for long-term use. Our study got the approval of the Research Ethics Committee of First People's Hospital of Taizhou Affiliated Wenzhou Medical University. All patients unanimously signed informed consent forms.

### 2.5. Cell Culture and Transfection

Human THCA cell lines (CAL-62, BCPAP, TPC-1, and 8505C) and human normal thyroid epithelial cell line (Nthy-ori 3-1) were acquired from ATCC (Rockville, USA). Cal-62 cells were cultured in Dulbecco's modified Eagle's medium (DMEM) with 10% fetal bovine serum (FBS), penicillin (50 units/mL; Gibco), and streptomycin (50 *μ*g/mL; Gibco) as previously described. BCPAP cells, TPC-1 cells, and human normal cell line Nthy-ori 3-1 were cultured in Roswell Park Memorial Institute 1640 (RPMI 1640) containing 10% FBS (Gibco, Rockville, MD, USA), 100 *μ*g/mL penicillin, and 0.1 mg/mL streptomycin. 8505C cells were cultured in Minimum Essential Medium (MEM) with 10% FBS, penicillin (50 units/mL; Gibco), and streptomycin (50 *μ*g/mL; Gibco). All cell lines were grown at 37°C in a 5% CO_2_ atmosphere. The complete sequence of NRXN2 was amplified from the THCA genome and then ligated lentiviral construct pcDNA3.1 (GenePharma, Shanghai, China). Final positive clones of OVER-NRXN2 were verified by sequencing. Lipofectamine 2000 (Invitrogen, USA) was utilized to transfect indicated plasmid into cells as the manual instructed.

### 2.6. Total RNA Extraction and Quantitative Real-Time PCR

Total RNA from tissues and cells was extracted using RNAiso Plus (Takara Biotechnology Co., Ltd., Dalian, China). The whole RNA was isolated referring to the instruction. Harvested RNA was then subjected to qRT-PCR analysis. Briefly, cDNA was reversely transcribed from RNA utilizing the Reverse Transcriptase kit as the protocols depicted (Vazyme, China). Quantification of NRXN2 mRNA was run utilizing the SYBR Green Master Kit (Vazyme, China) on the ABI 7900HT sequence detection machine (Bio-Rad, CA, USA). Glyceraldehyde-3-phosphate dehydrogenase (GAPDH) was an internal reference and was utilized to normalize NRXN2 mRNA expression. The primer of NRXN2 and GAPDH was synthesized and purchased from GenePharma. The primer sequences were as follows: NRXN2, forward 5′-CAGCACGAGGATGGATCGC-3′ and reverse 5′-GCCCACGTTAAAGATCACCCC-3′. GAPDH was forward 5′-GGAGCGAGATCCCTCCAAAAT-3′ and reverse 5′-GGCTGTTGTCATACTTCTCATGG-3′.

### 2.7. Proliferation Assay

The CCK-8 Kit was taken to conduct cell proliferation (Beyotime, Shanghai, China). 2 × 10^3^ cells per well were inoculated in a 96-well plate in triplicate. Cells in each well were incubated with 10 *μ*L CCK-8 solution for 2 h at 37°C. The OD value of 450 nm was measured by absorbance reader MB-580 (HEALES, Shenzhen, China).

### 2.8. Transwell Assay

The Transwell assay was conducted utilizing Transwell chambers (8 *μ*m pore size, Corning, NY, USA) and matrigel (BD Biosciences, USA) to assess the metastatic capability of THCA cells *in vitro*. 5 × 10^4^ cells in each well were seeded into the upper chamber in a DMEM medium with 1% FBS. 600 *μ*L DMEM medium with 10% FBS was added into the lower chamber. At 24 h postincubation, the cells remaining in the upper chamber were removed with the use of wet cotton sticks. And cells in the down chamber were fixed and stained with DAPI. Then, the number of cells was monitored by a fluorescent inverted microscope (Mshot, Guangzhou, China).

### 2.9. Statistical Analysis

All represented data were shown as the mean ± SD of three separate experiments. SPSS 17.0 (Chicago, IL, USA) was employed to analyze the difference of data. ^∗^*P* < 0.05 indicated a statistically significant difference.

## 3. Results

### 3.1. Assessment of the Association between NRXN2 Expression and Clinicopathological Features

First, we explored the relationship between NRXN2 expression and the clinicopathological characteristics of THCA patients.  Figure 2 demonstrates that NRXN2 expression displayed a negative correlation with nodal metastasis status of THCA (Figure 2(a)) but exhibited a positive association with the age of patients (Figure 2(b)). N1 of THCA presented a lower expression level of NRXN2 (Figure 2(a)). No obvious difference in NRXN2 expression was shown between male patients and female patients with THCA (Figure 2(c)). NRXN2 expression in each grade of THCA samples was lower than that in normal samples (Figure 2(d)). In summary, NRXN2 was a possible biomarker for THCA patients.

### 3.2. NRXN2 Was Correlated with Tumor-Infiltrating Immune Cells in THCA

We validated the relationship between NRXN2 expression and immune cells in THCA. The data revealed that NRXN2 expression was greatly associated with the macrophage M0 (Figure 1(a)), and its expression might be related to the weakened antitumor function of specific immune cells, especially by modulating macrophages to participate in the response of immune cells in the microenvironment of neoplasm. In light of the median level of NRXN2, patients with THCA were classified into high expression and low expression of NRXN2 in two groups.

### 3.3. Elevated Expression of NRXN2 in THCA

TCGA database was taken to detect NRXN2 expression levels in the tissues of THCA. Our data showed that NRXN2 expression in primary neoplasm tissues was significantly lower relative to that in normal tissues (Figure 1(b)). Overall, the results showed that NRXN2 expression in the tissues of THCA was lower compared to that in normal tissues.

### 3.4. NRXN2-Related Signaling Pathways in THCA

In order to further study the probable role of NRXN2 in the tumorigenesis of THCA, important genes associated with NRXN2 were selected for pathway enrichment analysis.  Figure 3(a) depicts a summary of the enrichment results. Significantly enriched terms were phase 2-plateau phase, NCAM signaling for neurite out-growth, Ca^2+^ pathway, NCAM1 interactions, beta-catenin independent WNT signaling, integration of energy metabolism, regulation of insulin secretion, cardiac conduction, muscle contraction, and neuronal system.

In addition, we used data in TCGA database to identify genes related to NRXN2 and predicted the signal pathways of NRXN2-associated genes. The results showed that a total of 20 important genes linked to NRXN2 were identified, including APBA2, GNA14, ABCC8, PRKCA, PRKACB, LRFN1, KCNJ8, ALDH2, KCNAB1, ITPR1, CACNB2, CACNB4, LMOD1, KCNE4, NPPC, KCNIP3, RYR2, and COL6A6. All these genes were related to the neuronal system, insulin secretion modulation, energy metabolism integration, muscle contraction, cardiac conduction, and NCAM1 interactions (Figure 3(b)).

### 3.5. NRXN2 Expression Was Downregulated in THCA

Figure 4(a) presents that, in comparison with adjacent normal tissues, the expression of NRXN2 mRNA was largely reduced in 35 paired tissues of THCA patients (*P* < 0.05). Besides, Figure 4(b) demonstrates a decreased expression of NRXN2 mRNA in CAL-62, BCPAP, TPC-1, and 8505C THCA cell lines, compared to that in human normal thyroid epithelial cell line (Nthy-ori 3-1) (*P* < 0.05). Our results implied that NRXN2 was probably implicated in THCA initiation and development.

### 3.6. NRXN2 Suppressed THCA Cell Proliferation

The CCK-8 assay was exploited to evaluate the impacts of NRXN2 on the proliferation of NRXN2-overexpressed THCA cells. We designed OVER-NRXN2 expression cassettes for overexpressing NRXN2. Our data exposed that OVER-NRXN2 had a high overexpression efficiency. NRXN2 was obviously overexpressed by transfection with OVER-NRXN2 in CAL-62 and TPC-1 cells (*P* < 0.001, Figures 4(c) and 4(d)). Overexpressing NRXN2 greatly retarded THCA cell proliferation (*P* < 0.05, Figures 4(e) and 4(f)).

### 3.7. NRXN2 Decreased Cell Metastasis in THCA Cells

We performed the Transwell assay to verify if NRXN2 could regulate THCA cell migration and invasion *in vitro*. After overexpressing NRXN2 in CAL-62 and TPC1 cells, we conducted cell migration and invasion assays. The result showed that the number of the adhered cell on the lower chamber membrane surface was significantly decreased compared to the control group (Figures 5(a)–5(h)). These results indicated that NRXN2 could suppress THCA cell metastasis.

## 4. Discussion

NRXN1, NRXN2, and NRXN3 are three important genes of NRXNs, which is a group of presynaptic unipath transmembrane proteins and functions as the organizers of synapse in mammals. The mutations of the NRXN2 gene were displayed in ASD, schizophrenia, ID, and other several neuropsychiatric disorders [7]. Considering the reports mentioned above, they paved the way for indicating that NRXN2 exerted a direct or indirect impact on human diseases. Nevertheless, it is yet elusive towards the roles of NRXN2 in the development of carcinoma.

The data from TCGA database revealed that NRXN2 expression in the tissues of THCA was lower than that in nontumor tissues. Similarly, NRXN2 expression in clinical samples of THCA was greatly lower relative to that of normal tissues. Many reports indicated that NRXN2 was a crucial factor in multiple diseases [11]. NRXN2 was reported to modulate NLRP3 in AD brain regions to affect Alzheimer's disease [12]. Another research reported that NRXN2 would modulate GAP43 and CASK in early cortical synaptogenesis which was diverse with NRXN1 and NRXN3 [13]. Besides, NRXN2 was also determined to join in the sex-differential DNA methylation and associated network [14].

In order to study the molecular function and potential mechanism of NRXN2 in the tumorigenesis of THCA, we conducted pathway enrichment analysis and identified 10 significant enrichment pathways. Then, we further identified 20 NRXN2-related genes. The signaling pathways of NRXN2-associated genes were mainly involved in the neuronal system, regulation of insulin secretion, integration of energy metabolism, muscle contraction, cardiac conduction, and NCAM1 interactions. The nervous system is seen as the tissue affected by cancer and as a channel for the spread of cancer pain and perineural invasion [15]. It has been reported that NRXN2 is one of the three human neurotoxin genes [7]. Inappropriate insulin secretion under low plasma glucose levels can cause severe and persistent hypoglycemia in newborns and children, leading to hyperinsulinemic hypoglycemia (HH) [16]. According to reports, energy metabolism is a core feature of tumor cells, and cancer cells must produce enough ATP to meet the energy requirements of overactive mRNA translation [17]. Exercise training is a prospective intervention strategy for preventing and treating carcinoma cachexia [18]. Patients with breast cancer presented obvious muscle strength disorders before and after anticancer treatment [19]. NRXN2 may participate in the tumorigenesis and development of cancer through these pathways, but there are few reports on the molecular function and potential mechanism of NRXN2 in cancer [20]. In addition, we found that NRXN2 was related to the weakened antitumor function of specific immune cells. This research provides a new direction for the research of NRXN2.

In previous reports, we found that there were a few studies on the role of NRXN2 in tumors. Additionally, we have not found any articles discussing the effect of NRXN2 on THCA. As a protein related to nerve cells, NRXN2 is related to many brain diseases [21]. In this study, we explored that NRXN2 was related to the formation of thyroid tumors and confirmed our hypothesis through a series of experiments. We carried out corresponding experiments to ascertain NRXN2's function in THCA in vitro. We believed that NRXN2 inhibited tumor progression by exerting proliferation and metastasis inhibitory effects in THCA. There are some limitations to this study. In the future study, we will further investigate the clinical significance and prognostic value of NRXN2 in THCA and conduct Western Blot experiment and animal model experiment on the basis of this study to further confirm the results of this study.

In conclusion, we proved the downregulation of NRXN2 in THCA and identified key genes related to NRXN2. Through KEGG, we analyzed the molecular function of NRXN2 in thyroid carcinogenesis. Our data revealed that lowly expressed NRXN2 in THCA took on an association with clinicopathological parameters and overall survival. NRXN2 expression was closely related to the antitumor function of specific immune cells, especially macrophage M0. All of our findings demonstrate that NRXN2 inhibited THCA cell proliferation, migration, and invasion *in vitro*. NRXN2 functions as a tumor suppressor gene and could serve as a novel target for THCA therapy. It might be a promising prognostic and therapeutic target in THCA.

## Figures and Tables

**Figure 1:** NRXN2 was correlated with tumor-infiltrating immune cells in THCA.

**Figure 2:** Assessment of the association between NRXN2 expression and clinicopathological features. (a–d) Data from TCGA: analysis of the association between NRXN2 expression and the nodal metastasis status, age, gender, and individual carcinoma stage of THCA patients.

**Figure 3:** NRXN2-related signaling pathways in THCA.

**Figure 4:** NRXN2 expression was downregulated in THCA. (a) Differences in NRXN2 expression between 35 THCA tissues and matched adjacent tissues. (b) Differences in NRXN2 expression between 4 different THCA cell lines (CAL-62, BCPAP, TPC-1, and 8505C) and human thyroid cell lines (Nthy-ori 3-1). (c, d) Determination of NRXN2 expression level in OVER-NRXN2 transfected TPC1 cell line and OVER-NRXN2 transfected CAL-62 cell line. (e, f) CCK-8 analysis of the influence of NRXN2 overexpression on TPC1 cell proliferation, CAL-62 cell proliferation. ^∗^*P* < 0.05 and ^∗∗∗^*P* < 0.001.

**Figure 5:** NRXN2 decreased cell metastasis in THCA cells. (a, b) Transwell assay analysis of the impacts of NRXN2 overexpression on TPC1 cell invasion. (c, d) Transwell assay analysis of the impacts of NRXN2 overexpression on TPC1 cell migration. (e, f) Transwell assay analysis of the impacts of NRXN2 overexpression on CAL-62 cell invasion. (g, h) Transwell assay analysis of the impacts of NRXN2 overexpression on CAL-62 cell migration. ^∗^*P* < 0.05.

## Data Availability

The datasets used and/or analyzed during the current study are available from the corresponding author on reasonable request.
